The article "A Case Study of the Famous Fantasia under the Development Variation Environment Monitoring to Analyze the Characteristics of the Composition of the Suite" was retracted in 2023. Reasons: signs of a paper mill; suspected computer-generated content; unreliable results or conclusions; concerns about the data.

# A Case Study of the Famous Fantasia under the Development Variation Environment Monitoring to Analyze the Characteristics of the Composition of the Suite

**DOI:** 10.1155/2022/7135360

**Published:** 2022-10-04

**Authors:** Yanan He, Qin Kang

**Affiliations:** School of Music, Hefei Normal University, Hefei, 230001 Anhui, China

## Abstract

In order to better grasp the quintessence of Brahms's suite-style piano suite and guide researchers and music creators, this thesis takes Brahms's late representative work Fantasia Op.116 as the research object and attempts based on the perspective of environmental monitoring of development and changes to analyze creative individuality in his seven works as well as the unity of the whole structure under the “developing variation” through elaborating the theory of “developing variation,” the creative features of works in Fantasia Op.116, and the unity of the materials under the “developing variation” from the perspective of creative techniques. The thesis finds that, on the one hand, Brahms used pitch interval structural capacity, nontraditional harmony, personalized rhythmic counterpoint, and prose structure and other specific variation techniques, embodying individuation differences and expanding the techniques used in the classical period; on the other hand, he changed, derived, and extended the theme motivation in works, specifically embodying the using of “developing variation” in his seven works, which solves the problems of unity and interconnectedness among works and provides inspirations for the creation of piano suites by later composers.

## 1. Introduction

In a “Radio Talk Marking the Centenary of Brahms's Birth” in 1933, Schoenberg positioned Brahms as a “progressive,” and since then, Schoenberg has modified the perception that western academics have of Brahms's work as a “conservative.” The works of Brahms were then reexamined and repositioned by Western academics. Since the 1980s, Chinese academics have also given Brahms's work more consideration. Based on the radio interview, Schoenberg wrote the article Brahms the Progressive [1], which established the growing variations as Brahms's fundamental musical technique and the basis for subsequent research on his compositions. Scholars were also drawn to Brahms's works, particularly in the 19th century when pianist suites were in demand. Research centred on creating variations, particularly the aspect of “unity” and how it permeates the entire work. Regarding “multi-piece” suites, these elements were the most significant aspects of Brahms's application of the idea of developing variation, which led to a lot of research and studies on the subject. Aside from that, was the development of Brahms's suite centred on accentuating the various qualities? In light of this, the author uses Fantasia, Op.116, a composition that might illustrate Brahms's innovation in later works, as an illustration to examine the variations between the individual pieces in a suite. What problems does the composer have to address in each piece? Or to put it another way, how can you separate out each work's traits and group these disparate pieces into a cohesive suite? What aspects of a composer's original thinking can be seen in a piece? Through the aforementioned inquiries, the study seeks to offer a fresh perspective on how Brahms's piano suites came to be, as well as some theoretical direction for other researchers working in this area.

## 2. Interpretation of Brahms's “Developing Variation”

Brahms is one of the most representative composers of the romantic period. Developing variation, being Brahms's core technique in music creation, has ascribed much attention by Schoenberg and attracted extensive attention and in-depth research from scholars at home and abroad. In fact, the concept was first put forward by Schoenberg in Bach1 in 1950, based on the contrast with polyphonic music, as a writing technique or composing philosophy relevant to the homophonic music style. The writing was then collected in Style and Idea (Arnold Schoenberg, “Bach”: Style and Idea, London: Great Britain by W &J Macay Limeted, 1975, p161). The original text is as follows:

The material of homophonic-melodic music, or music with a core theme supported by and based on harmony, is created by what I refer to as the development of variation. To elaborate on the piece's main theme, this means that changing the characteristics of a basic unit results in all the formulations that offer fluidity, contrasts, diversity, logic, and unity on the one hand, and character, mood, expression, and always-needed differentiation on the other.

The identical idea was put forth by Schoenberg in the motive chapter of his book Fundamentals of Music Composition. [2] Here is the original text:

The kind of music known as “growing variety” is homophonic. This indicates that there is something that may be compared to growth or development in the series of motive-forms generated by variation of the underlying motive. However, modifications to the subordinate meaning have just a limited embellishing impact and no specific repercussions. Variants are what we call such alterations.

Though being a core technique in Brahms's creation, the “developing variation” proposed by Schoenberg was, in the first place, a composing technique related to homophonic music development. In Brahms the Progressive, Schoenberg made excellent interpretation of the specific application of developing variation through analysis of Brahms's String Quartet Op. 51 No.2 in A minor.

Schoenberg did not, however, define “evolving variety” in the original text, which left some room for further research. Scholars continue to develop and enrich pertinent research in light of Schoenberg's analysis:

As shown in Table 1, in Brahms and the Principle of Developing Variation, foreign scholar Walter Frisch further expounded on Schoenberg's interpretation of developing variation from a more macroscopic perspective, believing that the developing variation not only is used to form the motive and theme but also was expanded into the usage of harmony, musical form and rhythm, integrating the different themes that run through several movements. A similar view could also be found in Michael Musgrave's Schoenberg's Brahm, in which he mentioned developing variation in the third part from the perspective of an outsider, analyzing Schoenberg's understandings of developing variation in Brahms's works. Based on this theory, the remaining four master's thesis and doctoral dissertations expanded the scope of their research, explaining the specific application of developing variation in Brahms's organ works, scherzos, piano quintet Op.34, and early piano works.

Four papers by Chinese scholars with detailed discussions on developing variation could also be found: (1) Yuan Lijun's Brahms in the Eyes of Arnold Schoenberg, published in the 2nd issue of the Journal of Tianjin Conservatory of Music (Sounds of Nature) in 2009; (2) Shanghai Conservatory of Music musicology major Zhou Weijuan's doctoral dissertation-On Innovation of Brahms Music; (3) Central Conservatory of Music musicology major Li Xin's master's thesis, Brahms's Principle of Developing Variation- A Case Study of Symphony No.4; and (4) the master's thesis of The Mengheng of Xi'an Conservatory of Music, The Neglected “Innovation” of “Tradition”-A Study of Principle of Developing Variation in Brahms's Third Symphony. Yuan Lijun first analyzed Schoenberg's understandings of the characteristics of Brahms's creation from the perspective of an outsider, including several related concepts, such as developing variation, “basic shape,” music prose, “feature,” and interval complex. Zhou Weijuan, Li Xin, and He Mengheng combed through the origin and development of the word “developing variation” from the diachronic aspect of music theory development with Schoenberg's understandings of Brahms's principle of developing variation as foundation and integrated other scholars' research to conduct in-depth explanations and summaries. The three scholars put forward similar views on the definition of developing variation, which includes two meanings: first, “developing” means the stability and unity of some core materials; and “variation” is the defining word of the term, which leads to the unique characteristic of the work. It also refers to the continuous derivation of new materials in the process of theme construction and development, completed by variations of interval, rhythm, harmony, and other factors, which not only could be used in different parts of the work but also run through the whole work, so that the music could head forward. It could be seen that, in their analysis, the four authors all revolved around the unity of developing variation, which has obtained wide consensus among Chinese scholars, providing an effective reference for further studies of Brahms's music creation.

Piano suite is the key genre of Brahms's late-creation, with the problem of “unity” and “run through” as his crucial tasks. This could be exemplified by his representative, transitional, and conclusive work Fantasien Op.116, which has drawn the attention of foreign scholars. By consulting the CNKI and other information platforms, the author found that most foreign scholars focused on the techniques that occur in all of the 7 pieces of Op.116, which aim to maintain the integrity and consistency of the works. A rather pronounced paper is The Multi-piece in Brahms: Fantasien, Op.116, written by Dunsby Jonathan and published in Brahms: Biographical, Documentary and Analytical Studies [3]. The paper mainly discusses the key material composition, tonality structure, and other aspects of the general layout, so as to demonstrate the relevancy and the unity of piano suite structures in Brahms's work [4]. The paper Elements of Unity in Fantasies, Op.116 by Brahms by Thomas Owen also demonstrated the unity and the “run through” elements of Op.116 as a whole.

Chinese scholars made relatively fewer analyses on Brahms piano suites Op.116. In total, there are 6 master theses and 2 journal articles. Seven of them focused on the analysis of performance, while only 1 paper focused on the analysis of the technique (The master's thesis of Zhao Tong from Jilin College of the Arts: Research of Harmonic Analysis of Brahms's Late-Piano Suite Op.116-119). From the perspective of the use of harmony, Zhao Tong conducted a detailed study of harmony techniques in Brahms's late-piano suite Op.116-119 and discussed it from three aspects, including Brahms's life history, harmony vocabulary, and other characteristics, providing certain references to analyze the characteristics of Brahms's late-piano creations.

Thus, it is clear from the analysis above that there is still opportunity for Chinese academics to study Op.116. Although more in-depth and focused research has been conducted by foreign experts, this work focuses on a different topic. This essay tries to elaborate on the distinctive production qualities, features, and significance of each of the seven parts in the piano suite, in addition to the suite's unity and relevance, and the rationale behind its pairing.

## 3. An Analysis of Brahms's Fantasien Op.116

The piano suite Fantasien Op.116 encompasses 7 pieces of music with concise form, short structure and poetic temperament. Among them are three passionate romantic caprices and four introversive and deep yet sensitive intermezzos. The theme and structure development, the complex rhythm, the contrapuntal musical texture, and the unique harmony showcase Brahms's mature composing style. The overall structure of the seven pieces is shown in Table 2.

### 3.1. No.1 Structural Forces of the Third Interval

For the first piece of the piano suite, Brahms used the sonata form common in the classical times to introduce his first Capriccio. Detailed illustration is provided in Figure 1 and Table 3.

At the beginning of theme A, Brahms used his favorite “descending third motive” (Brahms's Symphony No.4, for example, made full use of the third motive) and presented the work in chord texture. The bass part begins to respond since the third beat, forming an imitation. The vertical and horizontal third relation becomes an important structural factor of the theme, and the harmony formed is relatively simple, accompanied by rhythmic displacement, promoting the continuous development of music. Theme B used descending third motive to set up a harmony framework vertically for semitone motion. Theme C intensified the decomposition of the diminished seventh chord and strengthened the progression through octaves with rhythmic differences and contrary motion. The seventh-chord acoustic framework, which is primarily focused on the third relation, has allowed the work to remain cohesive even if the three themes with distinct qualities recurred throughout the suite. In addition, the passage played in 3/8 time, aside from the longa at the cadence, is typically made up of quavers and quarter notes, without the presence of beats of shorter span to provide a contrast or to advance the progression. These two very fundamental notes enable seamless transitions between triple time and duple time as well as adjustments in time according to accents. The upper and lower accents are placed on the first and third beats, respectively, of theme A, which begins in triple time and goes back two beats for imitation. Theme B is played in duple time and moves back one beat for imitation, so that the upper and lower accents are alternately stressed. Theme C returns to the triple time, with the upper and lower accents alternating with one beat moved back. The chord poured energy into the music, forming great tension and pushing the music forward. Finally, as shown in Figure 2, the third interval is also leading the whole work within the framework of the bass tone and tonality.

### 3.2. No.2 Distinctive Rhythm and Beat Counterpoint

The second intermezzo features “meditation” and is composed in rounded ternary form. “It genuinely restored Brahms's introspective style: a soft andante, almost like a Sarabande, with quiet and repeated cadence and minimal embellishment. The single episode and the ‘trio' are composed by broken octaves. The left hand pattern is supplied with subtle semitones” [2]. It could thus be concluded that the application of the main theme and motive is conducted in small range and is relatively simple. As shown in Table 4, in this sort of slow piece, Brahms used intricate rhythm, beat changes, and counterpoint to inject vitality to the rhythm as well as push the music forward.

The A section is played in 3/4 time with hemiola (2 : 3) to produce the counterpoint. The melody of the main theme used half note to form a slight pause and a subtle emphasis on the accent in the second beat. Repetition occurs after eight bars with simple embellishment on the previous half note to slightly accelerate the rhythm. In the middle section, Brahms adopted the same time signature-3/8-throughout the whole section, but the beats swing between triple time and duple time and form vertical and horizontal counterpoint, which is rather unique in design. The A section is shown in Figure 3.

From the above illustration, the first 5 passages are played in horizontal duple and triple time, which set up the basic ratio changes (2 : 3). The number of beats also multiplies accordingly. At the end, it retrogrades to the start to create a symmetric form (the last two passages could be seen as a prolongation of the longa). Vertically speaking, the upper and lower part has also form the ratio of 3 : 2 from the second beat, after which the accents of the lower part has formed counterpoint with the upper part at a misalignment of one beat's length until the second-to-last passage. It can be seen that Brahms flexibly applied hemiola 2 : 3 into beat changes and counterpoint, breaking through the traditional usage of rhythm and beat and the limitation of bar-line, so as to turn the irregular rhythm and the beats to good account and enrich the way to express rhythm and beats.

### 3.3. No.3 Special Harmony Technique

The third passionate “Fantasien” is also composed in rounded ternary form. The “wild” feature of the first and the last passage and the chorale-like heroism style of the middle section are in stark contrast. In this piece, Brahms adopted distinctive harmony techniques featuring unity, ambiguity, and symmetry. First of all, the splashing third chord reminded us of the descending third motive in the first piece. The “wild” passage is mainly composed of seventh chord materials formed by third motive, but with more structural expansion, for it not only creates melody and bass line in a horizontal fashion, but also shape chord in a vertical way. In its intricate development, the work has structure a multidimensional space that is vertical, horizontal and a space for dialogues, integrating and unifying vertically and horizontally the harmony, melody and bass. The piece is illustrated in Figure 4.

Secondly, the harmony framework in the exposition is regularly applied in the chord of the seventh (subdominant) of the two functional groups. As illustrated above, the time value-descending functional chord is developing through repetition and sequence (one s-D every two passage in the first eight passages; the frequency is reduced by twice in the last four passages), forming the sole stable tonic chord until the end. Prolonged avoidance of the tonic chord and the unstable acoustics of the seventh chord present an obscure and volatile condition. In classical time, this method is usually used for chord layout in the middle section. Placing the obscure and volatile chord at the very beginning of the piece has created a special characteristic. The same structural characteristic is also embodied in the seventh “Fantasien.” At last, the symmetric feature is also displayed in many aspects of the work. For instance, the general tonality layout of “g-BE-G-BE-g”; partially speaking, the tonality at the end of the two passages of the exposition is also symmetric; the tonality of the sequence part in the first passage (the last four bars in the above illustration) is g-A-B-g; the tonality of the sequence part in the second passage is g-#f-f-e-g; in terms of chord composition, while completing the chord progression, the last four bars of the above illustration also have the exact symmetric chord forms.

It could be concluded that the consistency, fuzziness, and symmetry of the chord have laid a unified basis for the music, as well as creating contrast, providing space for diversified musical emotions in different passages and forming rich and sound structural forces and the sense of forms.

### 3.4. No.4 The “Music Prose” Characteristic of “Developing Variation”

The fourth pastoral intermezzo is composed of three constantly changing music themes. It does not belong to the traditional trilogy style. Nor does it have recapitulations. Throughout the piece, Brahms adopted the technique of developing variation, which greatly guarantees the overall unity of the free form. The composition of the materials of the three themes is illustrated as Figure 5.

As can be seen from the example, the three thematic units are formed on the basis of the original motives—“a” (second) and “b” (third). Thematic unit A emphasizes the motive “a” (composed of the second), in which the dominant is raised by half a semitone. It plays the role of introduction and connection. Thematic unit B echoes with motive “a” in two parts. The inner voices lines are slightly extended through (b+c), and are further extended through material e+f in the second repetition (bar 5-9). Thematic unit C is the vertical combination and extension of c+f. In total, thematic unit a variation appears three times, and the materials of which gained slight extension through repetition of the motive “a.” Changes mainly happen in the aspect of tonality. As shown in Figure 6, the first variation (bar 32-36) made slight thematic extension in #g minor, the second variation in #C major, and the third back to original key E major.

The developing variation is carried out by the thematic units B and C, who both occur as imitative counterpoint or chord melodies in the middle lines. It is clear that Brahms's poetic utterances differ significantly from those of Chopin. Chopin's works frequently use stylistic devices including the tonic key declaration, extended lines, shifting rhythm, groups of grace notes, and rich chord application. However, Brahms uses the same strategies in a more restrained manner. Additionally, the piece is enhanced by the combination of his prose-like form, the straightforward musical theme, the multi-level melody, and the development and extension of the middle lines.

### 3.5. No.5 Unconventional Harmony Progression

The fifth intermezzo is of “andante con grazia ed intimissimo sentiment” and is also composed in the rounded ternary form. It could be seen from the score bellow that Brahms used relatively simple musical theme materials and texture. For the middle part, he used prolonged dominant, based on which the ascending third is “flowing” up and down to from imitation in the background of counterpoint. The exposition and the reprise are presented in columns of chords and “bare” intervals. The thematic materials of the second circumferential motive are included in the progression of chords and intervals, reminding us the thematic materials of the second intermezzo, as shown in Figure 7.

Brahms made some breakthroughs in the harmony progression of this work, which are mainly reflected in the direct collision of unsolved dissonance, parallel harmony progression with reduced function and the application of wrong notes. Firstly, each of the above chords is distributed in the upper and lower part in the form of inversion, forming interesting symmetry vertically (the third piece of Fantasien also has the horizontal symmetry chord structure). [5, 6] The next two dissonances have clear representation and direct collision, but the constituent notes hidden in them are rarely solved. At the same time, chords on the weak beats and the interval on the strong beats are changing the traditional metrical procedures in rhythm. In harmonic progression, Brahms used a series of ascending parallel harmony to accelerate the flow of music at a rate of exponential decline, as shown in Figure 8.

The first ten bats of the opening passage's theme melody statement are composed in a highly conventional style. A typical independent phrase (Satz) structure is created by cutting and combining musical elements that are introduced in the exposition and sequence. The in situ chord and the sixth chord are two different forms of the same chord that make up the lower harmonic section. These two chords are arranged ascending and parallelly to move the music along in step with the rhythm's decreasing frequency. The function and strength of harmony progression are somewhat diminished by the usage of parallel harmony. This method is widely used by romantic musicians to convey inner thoughts and natural scenery. This technique was used by Brahms, who focused on the lines while weakening the function by applying contrapuntal thinking to the parallel chords scattered throughout the upper and lower parts. The upper chord solver moves back one beat in the statement of the last four bars to become the next chord's dissonance at the same time. This chaining form enhances the shifts in musical colour by continuously introducing discord into the acoustics.

### 3.6. No.6 Intricate Counterpoint

As a composer who excels at counterpoint, Brahms used double counterpoint to set up the framework of this piece in rounded ternary form. As shown in Figure 9, the beautiful theme and melody are surrounded by the harmonic texture, with occasional changes to the soprano part and the bass part. A subordinate melody is also developing on the opposite direction, forming double counterpoint. It is particularly evident in the middle section. In the first seven bars, a progressive linear melody floats above the continuous imitation of the triplet rhythm. From the eighth bar, the triplet and the linear melody flow freely in the upper and lower part, forming also a double counterpoint. Compared with traditional counterpoint, Brahms is more restrained in part composition, more adventurous in harmony processing, and freer in the use of nonharmonic tones.

From the preceding score, it is clear that Brahms used homophonic harmony to depict the piece's polyphony and counterpoint. He introduced the piece with a theme melody that had a half-semitone increased dominant in the middle part, which served as a reminder of the fourth intermezzo's opening motive. Additionally, it illustrates Brahms's conservative approach to part processing. There are suspensions and appoggiaturas as a result of the many chromatic lines, which were eventually reconciled. Nonharmonic tones were frequently used in classical music's higher regions to evoke a sense of unease and the hope for a resolution. However, due to the chromatic lines in Brahms's composition, multiple suspensions and appoggiaturas appear in the upper part, along with appoggiaturas in the bass part, and were resolved in ascending minor second (as shown above). Finally, enharmonic change is employed to conduct contraposition of the distantly related key, highlighting the variations and contrasts of the acoustic colours while also making the chord more creative and intriguing. The counterpoint style is also integrated into the harmonic hues of the works from the second half of the 19th century using this harmony approach (as shown in Figure 10).

### 3.7. No.7 Comprehensive Reprise

The last piece of “Fantasien” still follows the passionate style of the previous pieces. The beginning is filled with the diminished seventh chord figure based on descending thirds, with the main characteristics being the unity of the chords and the inversion of the ternary form (as mentioned in the third piece). The middle section is composed of rounded ternary form. The two-against-three rhythm that almost vertically runs through the whole work is still the common technique used by Brahms. Generally speaking, the beats has integrated the rhythm of the former pieces in a horizontal fashion with frequent changes (2/4, 6/8, 2/4, 3/8, and 2/4). Besides, the broken chord texture freely converts in the upper and lower parts, forming a sort of alterations of the musical plane similar to double counterpoint. This is also the case in the fifth and the sixth intermezzos.

The toccata-like cadenza showcased its bridging role and paved the way for the reprise. The later part of the reprise transformed the broken diminished seventh chord figure into chord structure, bringing back the memories on the first piece, including the materials, rhythm and beats, and the triple and duple time, and forming a comprehensive reprise to successfully end the whole suite [7, 8].

In summary, the seven piano pieces enjoy different styles and are perfectly interpreted by Brahms in terms of interval, rhythm [9–12], harmony, structure, counterpoint and other techniques [13–16], among which the rhythm diversification [12, 17], counterpoint, functional harmony progression, and the music-prose style all display Brahms's inheritance and breakthrough of traditional composition techniques [18, 19]. As for piano suite consisting of several pieces, compared to the piano suites of other composers in the romantic period, Brahms tried to pursue characteristic differences, as well as integrate the relevancy of musical materials and the general tonality layout. In The multi-piece in Brahms: Fantasien Op.116, Jonathan Dunsby made excellent analysis on the relevancy and unity of musical materials in the work.

The two thematic materials were clearly separated by Jonathan Dunsby from the beginning of the first caprice, as seen in Figure 11, and he then demonstrated the evolving variation techniques, such as simple counterpoint, inversion, extension, and interpolation, in the following six pieces. These techniques are used throughout the “multi-piece” work to ensure the unity of the materials. For instance, the second and seventh pieces used straightforward counterpoint. The two primary components are presented inverted; the fourth, fifth, and sixth pieces included additional thematic materials that were based on the main theme's backbone lines and employed grace notes to amplify those materials.

Besides, the inner relevancy of the “multi-piece” tonal structure is also one of the main characteristics of Brahms's multi-pieces. This could be illustrated by Figure 12 in Jonathan Dunsby's paper.

The seven pieces are mainly composed of 4 different tonalities. The overall framework of tonality develops around d minor and the dominant key a major, forming a large functional framework of I-V-I tradition. The g minor and E major within the structure emphasize the tonic key and the dominant key through neighbor notes, especially during the long-time application in the middle part in e minor. The prolongation of the tonal center is a common technique of Brahms's to control the length of his works and also a crucial measure to strengthen the unity of the multi-piece. In Op.118, Brahms continued to attach importance to the unity of tonality, using alternating extension of the major and minor key of the same tonic and descending second sequence (for instance, a-A-g-f-F-be) to unify the whole work.

## 4. Conclusion

To sum up, Brahms made a good summary of his late life's creation with extremely simple forms, genres, and structures. First of all, Brahms made a good interpretation of the individual differences under the “developing variation” in pitch interval, rhythm, harmony, structure, and counterpoint from his seven piano pieces with different styles. Among them, the diversified rhythm, the counterpoint technology, weakening the functional harmony, and the musical prose structure also reflected Brahms's inheritance and breakthrough of traditional creation techniques.

Secondly, with regard to the piano suite, Brahms not only followed individual differences but also exploited the increasing variation on theme motivation in many pieces, in contrast to other composers' popular piano bagatelles throughout the romantic era. The entire structure of the pieces was able to reach perfect unity in this way. We can see that Brahms improved the connections between various works, so they were no longer just a collection of standalone pieces. He resolved the interdependence and unity between several works using material and tonal structure arrangement, which helped later composers when they were writing piano suites.

Last but not least, Brahms's “developing variation” based on precise pitch intervals or motor control modified the conventional pitch organisation that focused on tonal harmony and successfully addressed the issue that it was difficult to unite the motivation, melody, harmony, structural, and other factors in a piece when tonality was hazy and harmony function was attenuated. More crucially, Brahms's use of “developing variation” to organise pitches provided significant inspiration for later composers, particularly for Schoenberg.

## Figures and Tables

**Figure 1:** Sonata form of caprice.

**Figure 2:** Framework of the theme line and bass line and tonality layout.

**Figure 3:** Beat counterpoint.

**Figure 4:** Harmony analysis of the third “Caprice.”

**Figure 5:** Material analysis of the fourth “Intermezzo.”

**Figure 6:** Material analysis of the fourth “Intermezzo” material analysis of the fourth “Intermezzo.”

**Figure 7:** Material analysis of the fourth “Intermezzo.”

**Figure 8:** Frame of harmony.

**Figure 9:** Frame of harmony of the sixth “Intermezzo.”

**Figure 10:** Musical material analysis of Jonathan Dunsby.

**Figure 11:** Musical material analysis of Jonathan Dunsby.

**Figure 12:** Frame of tonal structure in Jonathan Dunsby's paper.

**Table 1:** Example of relevant studies.

Name	Paper	Date
Frisch, Walter	Brahms and the principle of the developing variation (University of California Berkeley)	1984
Michael Musgrave	Schoenberg's Brahms	1990
Larey Franklin	Developing variation, thematic transformation and motivic unity in the “quintet for piano and strings” Op. 34, by Johannes Brahms (University of Cincinnati)	1996
Landis, Raymond Eric	Developing variation in the chorale preludes for organ, opus 122 by Johannes Brahms (University of Cincinnati)	2001
Nie James Ian	“Developing variation” in Brahms's scherzos and scherzo substitutes (New York University)	2002
Nakatani Masafumi	The effect of the developing variation technique on Brahms's early piano solo works in the form of theme and variations (University of Miami)	2017

**(a):** 

Number	1			2			3			4
Name	Caprice			Intermezzo			Caprice			Intermezzo
Musical form	Sonata form			Single-trilogy form			Multiple trilogy form			Free form
Tonality	D-F	d-a-#c	BB-d	a	a-e-a-d-a	A-a	G	BE-G-BE	g	E-#g-#c-#g-E-#c-E
Tempo	Presto energico			Andante	Non troppo presto	Andante	Allegro passionato	Un poco Meno allegro	Tempo	Adagio
Main characteristic	The structural forces of the third interval			Special rhythm and beat counterpoint			Special harmonic technique			Developing variation: music prose

**(b):** 

Number	5			6			7		
Name	Intermezzo			Intermezzo			Caprice		
Musical form	Rounded single trilogy			Single-trilogy form			Multiple-trilogy form		
Tonality	e-b-e	e: D--	a-G-F-e	E	#g	E	d	a	d
Tempo	Andante con graaia ed intimissimo sentimento			Andantino teneramente			Allegro agitato		
Main characteristic	Unconventional harmonic progression			Intricate double counterpoint			Comprehensive reprise		

**Table 3:** The whole piece is composed of three main themes.

	Theme A: Descending third sequence with broken chords (D-bB-G-E) Polyphonic imitative texture, parallel harmony progression	1-4 205-208
	Theme B: F major dominant chord is harmonically established; ascending chromatic in the bass and inner voices under the minor seventh chord frame	24-36
	Theme C: Broken chords texture; mainly with the diminished seventh chord; statement in F major	37-52

**Table 4:** Characteristic of beat and rhythm.

Bar	A (1-18)	B (19-50)	A (51-86)
Beat	3/4	3/8	3/4
Rhythm	□	□.	□
Basic rhythm pattern			
Accent	The second beat	Mainly in the first beat; the longa is in the second beat	The second beat
Rhythm, beat counterpoint	2 : 3 (hemiola)	2 : 3	2 : 3

## Data Availability

The data used to support the findings of this study are available from the corresponding author upon request.
